The article "Diagnostic Value of MRI Combined with CXCR4 Expression Level in Lymph Node Metastasis Head and Neck Squamous Cell Carcinoma" was retracted in 2023. Reasons: unreliable results or conclusions; lack of ethics approval or compliance; concerns about the data; concerns about the peer review.

# Diagnostic Value of MRI Combined with CXCR4 Expression Level in Lymph Node Metastasis Head and Neck Squamous Cell Carcinoma

**DOI:** 10.1155/2022/4073918

**Published:** 2022-03-08

**Authors:** Jin Zhao, Xingde Li, Ming Wang, Fenghai Liu, Jingrun Wang

**Affiliations:** ^1^Department of Oncology, Cangzhou Central Hospital, Cangzhou, Hebei 061000, China; ^2^Department of Radiation Oncology, Cangzhou Central Hospital, Cangzhou, Hebei 061000, China; ^3^Department of Nuclear Magnetic Resonance, Cangzhou Central Hospital, Cangzhou, Hebei 061000, China

## Abstract

**Objective:**

To explore the diagnostic value of magnetic resonance imaging (MRI) combined with CXCR4 expression levels in lymph node metastasis of the head and neck squamous cell carcinoma (HNSCC).

**Methods:**

289 patients with HNSCC were divided into lymph node metastasis group (LNM group, *n* = 171) and non-LNM group (*n* = 118) according to the pathological examination results. MRI was used to scan the patient's lesions and cervical lymph nodes, and ADC was measured by MRI diffusion weighting imaging. The expression of CXCR4 in tumor tissues was detected by qRT-PCR. Logistic regression was used to analyze the risk factors of HNSCC lymph node metastasis. ROC curve was used to analyze the diagnostic effects of MRI, CXCR4, and MRI combined with CXCR4 on HNSCC lymph node metastasis.

**Results:**

Compared with the non-LNM group, patients in the LNM group had a lower degree of pathological differentiation, and the positive rate of TNM staging and vascular invasion was higher. The signal intensity of T1WI and T2WI were low intensity and high intensity, respectively, and the ADC value was significantly reduced. At the same time, the expression level of CXCR4 in the tumor tissues of the LNM group was also significantly increased. In addition, compared with MRI and CXCR4 used alone, MRI combined with CXCR4 has a higher predictive value.

**Conclusion:**

MRI has a good effect in demonstrating lymph node metastasis. CXCR4 is significantly upregulated in lymph node metastasis tumor tissue. The combination of the two can be used for clinical diagnosis of HNSCC lymph node metastasis.

## 1. Introduction

Malignant head and neck squamous cell carcinoma (HNSCC) are more common in China, accounting for about 5% of all malignant tumors in the human body [1]. They are mainly divided into three parts: oral and maxillofacial tumors, neck tumors, and otorhinolaryngology tumors. There are many primary sites and pathological types of these tumors at the top of systemic tumors [2, 3]. Smoking, alcohol, and HPV infection are the most important factors in the pathogenesis of the head and neck malignancies [4]. 90% of patients with the head and neck malignancies are 50–60 years old, mainly originating from the lymphatic tissue around the pharyngeal lymphatic ring or the squamous cells on the oropharyngeal mucosa. Due to a large amount of lymphatic tissue in the head and neck and abundant drainage, patients with HNSCC may have had one or more lymph node metastases at the time of diagnosis. At the same time, their early symptoms are mild and difficult to diagnose. Therefore, in most cases, only when the tumor is advanced or when the lymph nodes of the head and neck are found to have metastasized can the patient be diagnosed with malignant tumors of the head and neck.

The current clinical diagnosis of metastatic lymph nodes is often based on morphological criteria [5–7]. The diagnosis of HNSCC is usually based on routine histopathology [8]. Still, in recent years, magnetic resonance imaging (MRI) has also been increasingly used for the differential diagnosis of benign cervical and malignant lymph nodes. In imaging, a lymph node short diameter greater than 10 mm, central necrosis, annular enhancement, and extracapsular invasion are often used as the diagnosis basis for metastatic lymph nodes [9]. Among them, lymph node size is the most commonly used indicator in the diagnosis of metastatic lymph nodes. However, studies have found that the volume of many metastatic lymph nodes may also be within the normal range, and lymph nodes that have increased in volume may also be benign lymph nodes [10]. Therefore, using lymph node size as a criterion to distinguish between metastatic lymph nodes and benign lymph nodes in the neck has certain limitations.

The chemokine receptor CXCR4 is one of the cytokine-like protein families (CXC, CX3C, CC, and C). It is abnormally expressed in a variety of malignant tumors. Abnormal overexpression of CXCR4 is critical for the survival, proliferation, angiogenesis, homing, and metastasis of tumors [11], and increased expression of CXCR4 is usually associated with poor prognosis of patients [12, 13]. Studies have confirmed that the CXCR4 is involved in the metastasis of HNSCC [14] . Katayama et al. [15] showed that CXCR4 expression was significantly increased in HNSCC patients with advanced neck status and distant metastases, and that downregulation of CXCR4 expression inhibited tumor metastasis and progression in HNSCC patients. Albert et al. [16] Also clarified that CXCR4 may be a biomarker for high metastasis in HNSCC. However, there is no study that combines CXCR4 expression with MRI analysis in HNSCC. However, no research has used CXCR4 as a diagnostic marker for HNSCC. Therefore, in order to facilitate the diagnosis of HNSCC and their metastatic lymph nodes, in this study, the expression of CXCR4 in HNSCC combined with MRI was applied to the diagnosis of HNSCC with lymph node metastasis, and its feasibility and diagnostic value were explored.

## 2. Materials and Methods

### 2.1. Research Subjects

A collection of 289 patients with HNSCC admitted to our hospital from June 2016 to June 2018 were divided into lymph node metastasis group (LNM group, *n* = 171) and non-lymph node metastasis group (non-LNM group, *n* = 118). All patients have signed an informed consent form, and the Cangzhou Central Hospital committee approved this study (2020-250-01(Z)).

### 2.2. Inclusion Criteria

(1) HNSCC were diagnosed by histopathological examination; (2) all patients were primary tumors and had not received radiotherapy or chemotherapy before; (3) all patients underwent head and neck lymphadenectomy followed by pathological examination; (4) receive head and neck MRI before surgery; (5) complete patient clinical data; and (6) all patients are aware of the research content and have signed informed consent.

### 2.3. Exclusion Criteria

(1) Suffering from other malignant tumors at the same time; (2) received chemotherapy, radiotherapy, and immunosuppressive drugs before surgery; (3) incomplete clinical treatment; (4) MRI examination contraindication patients; (5) serious diseases of vital organs such as the heart, liver, and kidney; and (6) pregnant and lactating women.

### 2.4. General Patient Information

General information of the patients was recorded as follows: age, gender, primary tumor site, tumor size, degree of pathological differentiation (high, low), CT category, CN category, TNM stage, vascular invasion (negative/positive), paraneural invasion (negative/positive).

### 2.5. MRI Examination

The Signa HDe 1.5 T superconducting MRI imager provided by GE was used to scan the neck cross section, coronal plane, and sagittal plane using conventional spin echo (SE). T1WI and T2WI modes and using NMR diffusion weighting imaging (DWI) to measure the apparent diffusion coefficient (ADC). More than 2 radiologists read the image, and the short axis diameter of the lymph node tissue, signal intensity (uniform/uneven), margin (regular/irregular), boundaries (clear/unclear), T1WI signal intensity (high intensity/equal intensity, low intensity), T2WI signal intensity (high intensity/equal intensity, low intensity), ADC value were recorded.

### 2.6. qRT-PCR

TRIZOL (Invitrogen, Carlsbad, CA, USA) was used to extract total RNA from tumor tissues. PrimeScript™ RT reagent Kit (TaKaRa, Tokyo, Japan) was used for reverse transcription of RNA into cDNA. The PCR reaction was performed according to the operating instructions of the SYBR Premix Ex Taq™ II (TaKaRa) kit. The reaction conditions were as follows: 95°C for 10 s, then 95°C for 5 s, 60°C for 10 s, 72°C for 10 s, at a total of 40 cycles with the final 72°C extensions done for 5 minutes. GAPDH was used as the internal reference. The 2^−*ΔΔ*Ct^ method was used to calculate the relative expression of genes. The primer sequences were shown as follows: CXCR4, 5′-CTCCTCTTTGTCATCACGCTTCC-3′ (forward) and 5′-GGATGAGGACACTGCTGTAGAG-3′ (reverse); GAPDH, 5′-GGAGCGAGATCCCTCCAAAAT-3′ (forward) and 5′-GGCTGTTGTCATACTTCTCATGG-3′ (reverse).

### 2.7. Single Factor and Multiple Factor Logistic Regression Analysis

Analyze the degree of tumor histopathological differentiation, TNM staging, vascular invasion, CXCR4 level; lymph node tissue short axis diameter, signal intensity, margin, boundaries, T2WI signal intensity, ADC value, and correlations with HNSCC lymph node metastasis. Variable assignment was shown in Table 1.

### 2.8. Statistical Analysis

The data were statistically processed using SPSS 21.0 software (SPSS Inc., Chicago, IL, USA). The count data were described by the number of cases and percentage (%), and the difference between two groups was tested by chi-square test. The measurement data are described by the mean ± standard deviation (SD), and comparison between the two groups were performed using Student's *t*-test. The receptor operating characteristic (ROC) curve was used to evaluate the diagnostic value of MRI and CXCR4 in HNSCC. *P* < 0.05 indicates a significant difference.

## 3. Results

### 3.1. General Information

The general information of the enrolled patients was shown in Table 2. There were no significant differences in age, gender, primary tumor site, tumor size, CT type, CN type, and paraneural invasion (negative/positive) among patients between the non-LNM group and the LNM group. At the same time, the degree of pathological differentiation of patients in the LNM group was lower than that in the non-LNM group. The LNM group was significantly reduced, and the TNM staging and vascular invasion positive rate were increased considerably.

### 3.2. MRI Imaging Findings of Lymphoid Tissues in Non-LNM Group and LNM Group

MRI scans were performed on two groups of patients with HNSCC. The results showed that the short axis diameter of the lymph node tissue in the LNM group was significantly increased compared with the non-LNM group. The signal intensity was uneven, and edges were irregular, the boundary was not clear. The signal intensity of T1WI and T2WI were low intensity and high intensity, respectively. The ADC value was significantly reduced (Table 3). MRI images (Figures 1(a)–1(d)) show the characteristics of lymph node metastasis in a patient with the head and neck cancer: lymph node tissue T1WI shows low signal intensity, T2WI shows high signal intensity, and showing lymph node enlargement; DWI showing high signal intensity in lymph nodes, and ADC showing a high-intensity signal, indicating that the diffusion of water molecules in the lymph nodes is limited.

### 3.3. High Expression of CXCR4 in HNSCC with Lymph Node Metastasis

Further examination of the expression of CXCR4 in tumor tissues using qRT-PCR was done. The results showed that compared with the non-LNM group, the expression level of CXCR4 in the tumor tissues of the LNM group increased significantly (Figure 2).

### 3.4. MRI Imaging Indicators and CXCR4 Expression Are Significantly Correlated with Lymph Node Metastasis of HNSCC

The single-factor and multi-factor analysis of risk factors for lymph node metastasis showed that tumor tissue TNM staging, vascular invasion, and high CXCR4 levels; lymph node tissue short axis diameter, signal intensity, T2WI signal intensity, and ADC values are all related to HNSCC lymph node metastasis. There was no significant correlation between the degree of pathological differentiation, the margins and boundaries of lymph node tissue, and lymph node metastasis (Table 4).

### 3.5. The Combined Use of MRI and CXCR4 Enhances the Ability to Predict Lymphatic Metastasis of HNSCC

In order to further evaluate the diagnostic ability of MRI and CXCR4 for lymphatic metastasis of HNSCC, we performed ROC curve analysis. The results showed that the expression of CXCR4 (AUC = 0.9185) and MRI (AUC = 0.9335) alone predicted tumor ability and was lower than the expression of CXCR4 in combination with MRI (AUC = 0.9605) (Figure 3). This result suggests that the combination of CXCR4 and MRI may be a new method for diagnosing lymphatic metastasis of HNSCC.

## 4. Discussion

HNSCC is the fifth most common tumors worldwide, with about 500,000 new cases each year, of which more than 300,000 people die [17]. The main histological type of HNSCC is squamous cell carcinoma [18], and most patients are already in the advanced stage at the time of diagnosis, so the mortality rate is high. MRI is a commonly used and vital clinical imaging diagnostic method. It has the characteristics of multiparameter imaging, mainly including diffusion weighted imaging, diffusion tensor imaging, perfusion weighted imaging, dynamic enhancement scanning, magnetic resonance spectroscopy, and blood oxygen level dependent imaging. This can prompt information about the anatomical structure and functional imaging and provide more information about lymph nodes and their surrounding tissues [19]. It has been gradually used in the diagnosis of a variety of malignant tumors and their lymph node metastasis and has good diagnostic performance [20]. Diffusion weighted imaging is a sequence in MRI, which can reflect the diffusion and movement of water molecules in the organism and provide information on cell integrity and pathology. The apparent diffusion coefficient ADC value of the tissue reflects the comprehensive microscopic movement of the molecule. By quantitatively measuring the ADC value, it can reflect the diffusion characteristics of the molecule and indirectly reflect the change of the microstructure of the tissue [21]. This study mainly used two functional imaging methods, diffusion weighted imaging and dynamic enhanced scanning. We found that the short axis diameter, signal intensity, margin, boundary, T2WI signal intensity, and ADC values of the lymph node tissue in the LNM group were significantly different than those in the non-LNM group. This indicates that MRI has a good role in diagnosing HNSCC with or without lymphatic metastasis. For previous studies' preoperative staging of HNSCC, high-resolution MRI images were the mainstays, combined with fat suppression or ordinary enhanced scanning for observation. However, for patients who do not provide clinical history or early-stage small tumors, MRI images alone often cannot clearly display the area of interest which affects the staging judgment. Therefore, further exploration of biomolecular markers combined with MRI can improve the accuracy of the diagnosis of HNSCC with lymph node metastasis.

The metastasis of tumor cells is similar to that of normal cells and is regulated by chemokine receptors and their receptors, growth factors, adhesion molecules, and interstitial metalloproteinases. An increasing number of studies have shown that CXCR4 is the main chemokine receptor for tumor cell migration, and its expression level is positively correlated with the metastasis rate of tumor cells [22]. Tamamura et al. [23] first found that in a mouse model of breast cancer metastasis, injection of CXCR4 receptor inhibitors can significantly reduce the rate of breast cancer cell metastasis. Luo et al. [24] found that CXCR4 is overexpressed in laryngeal squamous cell carcinoma and can promote the proliferation and metastasis of cancer cells. In hematological malignancies and solid tumors, the overexpression of CXCR4 on the cell surface has also been shown to increase tumor cell survival and chemotherapy resistance and promote tumor cells to metastasize to organs [25]. CXCR4 is the main regulation axis of tumor cell migration [26]. In this study, we found that compared with the non-LNM group, the expression of CXCR4 in the tissues of the LNM group was significantly increased, which is consistent with previous studies and is associated with lymph node metastasis. In the ROC curve, we found that the diagnostic efficiency of CXCR4 alone is lower than that of MRI alone, but MRI combined with CXCR4 has the highest efficiency in diagnosing head and neck lymph node metastasis, which provides a new idea for the clinical diagnosis of HNSCC lymph node metastasis.

## 5. Conclusion

In summary, we first applied MRI and CXCR4 to the diagnosis of lymph node metastasis of HNSCC and found that MRI combined with CXCR4 can improve the diagnosis of lymph node metastasis of HNSCC. This can provide new ideas for preliminary clinical assessment of lymph node metastasis or prognosis of tumors.

## Figures and Tables

**Figure 1:** MRI image of a HNSCC patient with lymph node metastasis. (a) Patient T1WI weighted mode scan; (b) Patient T2WI weighted mode scan; (c) Patient DWI weighted mode scan image; and (d) Patient ADC image.

**Figure 2:** The expression level of CXCR4 in the tumor tissues of the two groups of patients. ^∗∗∗^*P* < 0.001 vs. Non-LMN group.

**Figure 3:** ROC curve of HNSCC lymphatic metastasis prediction characteristics.

**Table 1:** Assignment of variables.

Variable name	Assignment situation
Pathological differentiation degree	Low level = 0; high level = 1
TMN staging	Phase 2 = 2; phase 3 = 3; phase 4 = 4
Vascular invasion	Negative = 0; positive = 1
CXCR4 expression levels	Continuous variable
Short axis diameter	<5 = 1; ≥5 = 2
Signal strength	Uneven = 1; uniform = 2
Margin	Irregular = 1; regular = 2
Boundaries	Unclear = 1; clear = 2
T1WI signal intensity	Low intensity = 1; high intensity = 2
T2WI signal intensity	Low intensity = 1; high intensity = 2
ADC	Continuous variable

**Table 2:** Comparison of baseline related data between the two groups of patients.

Item	LNM group (*n* = 171)	Non-LNM group (*n* = 118)	*T*/*χ*^2^	*P*
Age	61.74 ± 6.65	60.47 ± 6.75	1.586*^Δ^*	0.114
Gender				
Male	69	49	0.040	0.842
Female	102	69		
Primary tumor site				
Head	73	56	0.642	0.423
Neck	98	62		
Tumor size				
<5	58	44	0.347	0.556
≥5	113	74		
CT type				
2	110	73	0.216	0.898
3	20	14		
4	41	31		
CN type				
Negative	0	0	—	—
Positive	171	118		
Paraneural invasion				
Negative	52	40	0.392	0.531
Positive	119	78		
Degree of pathological differentiation				
Low	111	91	4.944	0.026
High	60	27		
TMN staging				
0	0	17	166.801	≤0.001
1	8	66		
2	46	31		
3	117	4		
Vascular invasion				
Negative	61	91	48.104	≤0.001
Positive	110	27		

*Δ*: is expressed to perform an independent sample *T*-test, and the statistic was chosen as *T*.

**Table 3:** Statistical analysis of imaging manifestations of the two groups of patients.

Item		LNM group (*n* = 171)	Non-LNM group (*n* = 118)	*T*/*χ*^2^	*P*
Short axis diameter	<5	37	93	92.228	≤0.001
	≥5	124	25		
Signal intensity	Uniform	38	99	106.523	≤0.001
	Uneven	133	19		
Margins	Regular	53	90	57.259	≤0.001
	Irregular	118	28		
Boundaries	Clear	48	89	62.794	≤0.001
	Unclear	123	29		
T1WI signal intensity	High intensity	64	48	0.311	0.577
	Low intensity	107	70		
T2WI signal intensity	High intensity	107	16	68.612	≤0.001
	Low intensity	64	102		
ADC value		0.84 ± 0.15	0.92 ± 0.84	−5.949*^Δ^*	≤0.001

*Δ*: is expressed to perform an independent sample *T*-test, and the statistic was chosen as *T*.

**Table 4:** Single-factor and multi-factor analysis of risk factors for lymphatic metastasis.

Factor	Classification	Single factor		Multi factor	
		HR (95% CI)	*P*	HR (95% CI)	*P*
Degree of pathological differentiation	Low/high	0.549 (0.322–0.934)	0.027	0.407 (0.123–1.347)	0.141
TMN Staging	2 stage/3 stage/4 stage	0.065 (0.036–0.117)	≤0.001	0.238 (0.111–0.507)	≤0.001
Vascular invasion	Negative/positive	0.165 (0.097–0.280)	≤0.001	19.983 (9.971–432.000)	≤0.001
CXCR4 expression levels	Continuous variable	0.847 (0.817–0.877)	≤0.001	0.665 (0.576–0.766)	≤0.001
Short axis diameter	<5/≥5	0.074 (0.042–0.132)	≤0.001	0.114 (0.047–0.280)	≤0.001
Signal strength	Uniform/uneven	18.237 (9.918–33.532)	≤0.001	5.512 (2.350–12.926)	≤0.001
Margins	Regular/irregular	7.156 (4.196–12.204)	≤0.001	0.763 (0.293–1.986)	0.579
Boundaries	Clear/unclear	7.864 (4.603–13.436)	≤0.001	1.410 (0.584–3.404)	0.444
T1W1 signal intensity	High intensity/low intensity	1.146 (0.709–1.854)	0.577	—	—
T2W1 signal intensity	High intensity/low intensity	0.094 (0.051–0.173)	≤0.001	0.311 (0.137–0.708)	0.005
ADC	Continuous variable	201.622 (24.793–1639.665)	≤0.001	3597.151 (111.264–116295.301)	**≤0.001**

## Data Availability

The data used to support the findings of this study are available from the corresponding author upon request.
